# PDL241, a novel humanized monoclonal antibody, reveals CD319 as a therapeutic target for rheumatoid arthritis

**DOI:** 10.1186/ar4400

**Published:** 2013-12-04

**Authors:** Jacky Woo, Michel PM Vierboom, Hakju Kwon, Debra Chao, Shiming Ye, Jianmin Li, Karen Lin, Irene Tang, Nicole A Belmar, Taymar Hartman, Elia Breedveld, Vladimir Vexler, Bert A ‘t Hart, Debbie A Law, Gary C Starling

**Affiliations:** 1 AbbVie Biotherapeutics, 1500 Seaport Blvd, Redwood City, CA 94063, USA; 2 Department of Immunobiology, Biomedical Primate Research Centre, Rijswijk, The Netherlands; 3 Current Address: Gilead, Foster City, CA, USA; 4 Current Address: Coherus Biosciences, Redwood City, CA, USA; 5 Current Address: Merck, Palo Alto, CA, USA

## Abstract

**Introduction:**

Targeting the CD20 antigen has been a successful therapeutic intervention in the treatment of rheumatoid arthritis (RA). However, in some patients with an inadequate response to anti-CD20 therapy, a persistence of CD20^-^ plasmablasts is noted. The strong expression of CD319 on CD20^-^ plasmablast and plasma cell populations in RA synovium led to the investigation of the potential of CD319 as a therapeutic target.

**Methods:**

PDL241, a novel humanized IgG_1_ monoclonal antibody (mAb) to CD319, was generated and examined for its ability to inhibit immunoglobulin production from plasmablasts and plasma cells generated from peripheral blood mononuclear cells (PBMC) in the presence and absence of RA synovial fibroblasts (RA-SF). The *in vivo* activity of PDL241 was determined in a human PBMC transfer into NOD scid IL-2 gamma chain knockout (NSG) mouse model. Finally, the ability of PDL241 to ameliorate experimental arthritis was evaluated in a collagen-induced arthritis (CIA) model in rhesus monkeys.

**Results:**

PDL241 bound to plasmablasts and plasma cells but not naïve B cells. Consistent with the binding profile, PDL241 inhibited the production of IgM from *in vitro* PBMC cultures by the depletion of CD319^+^ plasmablasts and plasma cells but not B cells. The activity of PDL241 was dependent on an intact Fc portion of the IgG_1_ and mediated predominantly by natural killer cells. Inhibition of IgM production was also observed in the human PBMC transfer to NSG mouse model. Treatment of rhesus monkeys in a CIA model with PDL241 led to a significant inhibition of anti-collagen IgG and IgM antibodies. A beneficial effect on joint related parameters, including bone remodeling, histopathology, and joint swelling was also observed.

**Conclusions:**

The activity of PDL241 in both *in vitro* and *in vivo* models highlights the potential of CD319 as a therapeutic target in RA.

## Introduction

Rheumatoid arthritis (RA) is a chronic autoimmune disease marked by chronic pain and joint damage characterized by synovial inflammation and hyperplasia. The pathology of RA is complex, with many different cell subsets playing a role in the disease initiation and progression [1]. One of the defining features of the disease is the presence of auto-antibodies in the serum, including rheumatoid factor (RF) and antibodies directed against cyclic citrullinated peptide [2]. Disease modifying anti-rheumatic drugs (DMARDs) include those targeting the underlying immune processes that drive the pathology, including small molecule immunosuppressive agents and biologics. The most widely prescribed biologic agents are blockers of the TNF-α pathway. Patients who become refractory to anti-TNF therapy may be treated with agents that target the IL-6 pathway (tocilizumab, binding the IL-6 receptor), prevent T cell costimulation (abatacept, which binds CD80 and CD86 [3]) or deplete B cells from the circulation (anti-CD20 mAb rituximab [4]). The production of auto-antibodies by cells of the B cell lineage prompted the investigation of anti-B cell therapies for treatment of RA [5]. However, B cell depletion has also been reported to affect other functions, including their ability to stimulate T cell proliferation, produce cytokines and assist in the development of lymphoid tissue architecture [6]. Despite the tremendous progress in the treatment of RA, a substantial group of RA patients have inadequate responses to current therapies or have safety issues. The presence of late stage plasmablasts as a marker of resistance in active RA patients non-responsive to anti-CD20 therapy [7] illustrates the need for therapies targeted against plasmablasts and plasma cells. CD20 is not typically expressed by immunoglobulin (Ig)-producing plasmablasts [8]. To this end, we attempted to identify new targets for development of RA therapeutics that target plasmablasts. Previous studies have demonstrated the expression of the cell surface glycoprotein CD319 on plasma cells [9], which became the focus of the current study.

CD319 (SLAMF7, CS1, 19A24, novel Ly9, CRACC) is a 66 kDa glycoprotein member of the SLAM superfamily [10]. Members of the SLAM superfamily share a common structure consisting of a membrane proximal C-type Ig fold and a membrane distal V-type Ig fold. The cytoplasmic region of CD319 contains two immunoreceptor tyrosine-based switch motifs (ITSM), which bind to SH2-only adapter molecules Src homology 2 domain protein 1A/SLAM-associated protein (SAP) and EWS-activated transcript-2 (EAT-2) [11,12]. Phosphorylation of the tyrosine motifs leads to activation of downstream molecules including PLCγ1, PLCγ2 and PI3K kinases and modification of a variety of cell functions. As observed with other SLAM family members, CD319 engages in homophilic interactions which may potentiate cell activation [13]. Interestingly in the absence of EAT, CD319-CD319 interactions may exert a negative regulatory effect on natural killer (NK) cells [14]. Two CD319 transcripts have been identified in human NK cells, with a shorter form of CD319 (CD319-S) postulated to have a separate function from the longer form (CD319-L) due to its lack of ITSMs [15].

Expression of CD319 is restricted to cells of hematopoietic origin including plasma cells, resting NK cells, a subset of CD8^+^ T cells and plasmacytoid dendritic cells (DC), with minimal expression on resting B cells, resting CD4^+^ T cells and monocytes [9]. Upregulation of CD319 expression has been observed following activation of B cells, CD4^+^ T cells, monocyte-derived DC and monocytes [16] suggesting that CD319 may play a role in immune regulation. In support of this hypothesis, high CD319 expression has been observed on plasma cells or B cells from several disease indications including systemic lupus erythematosus [17], and the transformed cells in multiple myeloma [16] indicating the potential for CD319 as a therapeutic target for plasmablast and/or plasma cell-driven diseases. In this study, we investigated the expression of CD319 in RA tissues, and generated PDL241, a humanized monoclonal antibody (mAb), to target cells expressing CD319. CD319 was expressed on plasma cells in RA synovial tissues. PDL241 inhibited the production of immunoglobulins in an Fc-dependent manner *in vitro* by killing plasmablasts and plasma cells. Finally, PDL241 was tested for activity in a human-severe combined immunodeficiency (hu-SCID) mouse model of Ig production and a rhesus macaque model of collagen-induced arthritis (CIA). The data demonstrate the potential of CD319 as a therapeutic target in RA.

## Methods

### Immunohistochemistry analysis

Synovial tissues were obtained from 26 individuals with RA according to the approved protocol (PDL-011-04RA) reviewed by the Mayo Clinic Institutional Review Board. All patients gave their written informed consent after the risks and benefits of the study were explained. The 1G9 mAb, which recognizes an intracellular epitope of CD319 [9], was used to stain formalin fixed paraffin embedded (FFPE) tissues using an automated immunostainer (Dako North America, Carpinteria, CA, USA) with 3,3′-diaminobenzidine detection (Ventana Medical Systems, Tucson, AZ, USA). Double labeling studies were performed using 1G9 in combination with an anti-CD3, anti-CD20, anti-CD56 (LabVision, Fremont, CA, USA), anti-CD68 (Dako) and anti-CD138 (Invitrogen, Camarillo, CA, USA). VS38c mAb (Dako) was also used as a plasma cell marker. PDL241 was used to stain optimal cutting temperature (OCT) embedded frozen tissues from human or rhesus monkeys for immunohistochemistry (IHC) and immunofluorescence studies. AF488-conjugated streptavidin (Invitrogen) was used to detect PDL241 staining after prior incubation with biotinylated donkey anti-human Ab (Jackson ImmunoResearch Laboratories, Inc., West Grove, PA, USA). AF555 or AF594- conjugated anti-mouse or rabbit secondary Ab (Invitrogen) were used to detect other cell surface markers in a co-staining study. Slides were counter-stained with 4′,6-diamidino-2-phenylindole (DAPI) to visualize cell nuclei.

### Generation of PDL241

Female BALB/c mice (Taconic, Hudson, NY, USA) were immunized with purified CD319 protein and mAb were generated by fusing spleen cells to the NS0 fusion partner (American Type Culture Collection). Anti-CD319 specific mAb were identified using a variety of selection techniques including ELISA for CD319 protein, immunoblotting and flow cytometry analysis of CD319-expressing and CD319 non-expressing cell lines. The mouse parental mAb of PDL241 (m241) was selected for its ability to bind to CD319 protein from human and non-human primates (NHP). M241, a mouse IgG1, was chimerized to human IgG1 for initial functional characterization prior to humanization. Humanization of m241 was performed by the method of Queen *et al*. [18] and resulted in PDL241, which was engineered onto an IgG1 κ backbone with T250Q and M428L mutations in the Fc domain designed to extend the *in vivo* half-life via an enhanced binding to FcRn [19]. A FcR-binding deficient mutant of PDL241 (241-G2M3) was made by fusing the PDL241 variable domains to human IgG2M3 Fc domains [20]. F(ab)’2 fragments were produced by pepsin cleavage and purification on protein A. The negative control IgG1 mAb (cIgG1) for PDL241 used throughout this study was MSL109, a fully human anti-cytomegalovirus mAb [21]. Material for *in vivo* studies was produced in NS0 cells. All materials were tested for endotoxin (<0.02 EU/mg) and protein aggregation (<1%).

### Peripheral blood mononuclear cells

Peripheral blood mononuclear cells (PBMC) were obtained from the heparinized blood of normal volunteer donors (AbbVie Biotherapeutics or Stanford Blood Center, Palo Alto, CA, USA) by separation on 50 ml Leucosep™ tubes (Greiner Bio-one N.A. Inc., Monroe, NC, USA) or Ficoll-Paque Plus (GE Healthcare Lifesciences, Piscataway, NJ, USA). After two rounds of washes with PBS, PBMC were resuspended at 1 × 10^6^ cells/ml in R-10 media (Roswell Park Memorial Institute (RPMI) containing 10% heat inactivated FBS, 1X Pen/Strep, 20 mM HEPES).

### Cell staining and flow cytometry

To determine the phenotype of cells that were bound by PDL241, 2 × 10^6^ PBMC collected from healthy individuals were labeled for analysis of lymphocytes, while 1 × 10^6^ PBMC were used for analysis of plasma cells and dendritic cells. After the addition of Fc block (Miltenyi, Auburn, CA, USA), PBMC were incubated at 4°C for 30 minutes with fluorochrome-conjugated antibodies specific for cell surface markers CD3 (SK7 and SP34-2), CD4 (RPA-T4), CD8 (RPA-T8), CD56 (MY31), CD16 (3G8), CD14 (M5E2), CD19 (SJ25C1), CD27 (M-T271), CD38 (HB7), CD11c (B-ly6), CD123 (7G3), HLA-DR (L243), and lineage cocktail 1 (lin 1) (BD Bioscience, San Jose, CA, USA) and CD138 (B-B4, Miltenyi) with AF488 labeled PDL241. Cells were washed twice with PBS and then analyzed on a BD FACSCanto.novi Luc90 (AbbVie Biotherapeutics) is an anti-CD319 mAb that does not compete for CD319 binding with PDL241.

### Pokeweed mitogen-induced IgM production assay

PBMC (2 × 10^5^ in 200 μl) were treated with cIgG1 or PDL241 in the presence of 0.25 μg/ml pokeweed mitogen (PWM) (Sigma, St. Louis, MO, USA) in 96-well round bottom plates. At day 7, supernatants were harvested and the level of secreted IgM was measured using an Easy-Titer IgM assay kit (ICL Inc., Portland, OR, USA) according to the manufacturer’s instructions. In some experiments, NK cells or monocytes were depleted from PBMC by positive selection using RoboSep^®^ (STEMCELL Technologies, Vancouver, BC, Canada) according to the manufacturer’s instructions.

### Cell depletion experiments

PBMC (4 × 10^5^ in 200 μl) were treated with cIgG1, PDL241 or rituximab in 96-well round bottom plates. Following six days of culture at 37°C, cells were harvested and the absolute count of each PBMC subset was determined by flow cytometry. PBMC were incubated at 4°C for 20 minutes with fluorochrome-conjugated antibodies (CD3, CD19 and CD27) in 100 μl PBS after the addition of Fc blocker. Cells were washed once with PBS and resuspended in 130 μl PBS containing 30 μl of counting beads. Samples were then analyzed with a BD FACSCanto and absolute cell counts were calculated using the following equation:

$$\begin{array}{ll} \frac{\text{number of cell events}}{\text{number of bead events}}\times & \frac{\text{assigned bead count of the lot}\;\left(\text{beads}/30\mu l\right)}{\text{volume of sample}\;\left(\mu ,l\right)}\\ & \;=\;\text{concentrat}\mathrm{ion}\;\left(\text{cells}/\mu l\right) \end{array}$$

% live cells were calculated as % of absolute cell number of test mAb over cIgG1.

### Co-cultures of RA-synoviofibroblasts with PBMC

RA- synovial fibroblasts (SF) were purchased from Cell Applications, Inc (San Diego, CA, USA), and routinely maintained in synoviocyte growth medium (Cell Applications) at 37°C, 5% CO_2_. RA-SF (passage number >5) were seeded into 24-well plates at 6 × 10^4^ cells per well and allowed to reach confluence for 24 hours. PBMC (6 × 10^5^/well) were added to the confluent monolayers of RA-SF. The co-cultures were then treated with mAb (10 μg/ml) for seven days. At the end of the culture period, PBMC (suspension and adherent) were harvested by extensive washing followed by trypsin-ethylenediaminetetraacetic acid (EDTA). PBMC were washed once with fluorescence-activated cell sorting (FACS) buffer (PBS + 2% FBS), and subjected to FACS staining in FACS buffer containing cIgG1 or Luc90-FITC and IgD-PE; and CD38-PEcy7, CD27-APC, and CD19-APCcy7.

### HuSCID model of IgM production

Human PBMC (2 × 10^7^) were injected into the peritoneal cavity of six to eight week old NSG mice (NOD.Cg-Prkdcscid Il2rgtm1Wjl/SzJmice, The Jackson Laboratory, Bar Harbor, ME, USA) in 200 μl of PBS. For histological examination of human leukocyte cell surface markers, mice were sacrificed 14 days post PBMC transfer to assess the cell viability and the expression of CD319 on human T cells, B cells, NK cells and plasma cells in the spleens. Sections (5 μm) were cut from OCT-embedded frozen spleens for immunofluorescence analysis as described above. Plasma was obtained from blood samples by centrifugation, and stored at −20°C until the time of analysis. Human IgM levels were measured as described above. These studies were performed in compliance with the U.S. Department of Health and Human Services Guide for the Care and Use of Laboratory Animals under a PDL Biopharma/Facet Biotech IACUC-reviewed and approved protocol.

### CpG-driven IgM production in rhesus monkey PBMC

Rhesus PBMCs were isolated by Ficoll gradient separation from freshly drawn rhesus blood (California National Primate Research Center (Davis, CA, USA)). Cells were cultured in 96-well plates in R-10 medium. The TLR-9 agonist CpG-B DNA prototype ODN2006 was obtained from HyCult Biotech (Plymouth Meeting, PA, USA), and added to cultures at a concentration of 2.5 ug/ml. Cells were cultured for thirteen days, and the IgM levels in culture supernatants were determined by ELISA.

### Rhesus monkey collagen-induced arthritis study

In accordance with the Dutch law on animal experimentation, the study protocol and experimental procedures were reviewed and approved by the Experimental Animal Care and Use Committee of the Biomedical Primate Research Centre (BPRC) before the experiments started. Animals were purchased from the Animal Science Department of the BPRC in Rijswijk, The Netherlands. CIA-susceptible monkeys were seronegative for the dominant class I major histocompatibility complex resistance marker *Mamu-B26*[22,23]. The total study group comprised of 24 young adult, healthy rhesus monkeys (*Macaca mulatta*). During the study the monkeys were housed socially, where possible, in cages specifically designed to house NHP. The animals were offered a daily diet consisting of monkey food pellets (Hope Farms, Woerden, The Netherlands), fresh fruit and vegetables and bread. Drinking water was available *ad libitum*. Analgesic medication (Buprecare^®^, 0.3 mg/ml buprenorfine base; Schering-Plough B.V., Maarssen, The Netherlands) was given based on the assessment of the animal caretakers and BPRC’s veterinary staff (start and dosing increased or stopped on the basis of behavioral changes). The ulcerative skin lesions developing at the immunization sites were treated with wound spray (Acederm; Intervet, Boxmeer, The Netherlands) each time that an animal was sedated, in order to prevent infection. The study protocol was reviewed and approved by the BPRC Experimental Animal Care and Use Committee.

For induction of CIA, chicken type II collagen (chCII) was dissolved in 0.1 M acetic acid to a final concentration of 10 mg/ml and mixed with an equal volume of complete Freund’s adjuvant (CFA; DIFCO, Detroit, MI, USA). CIA was induced by injection of 1.0 ml emulsion (5 mg chCII/animal) into the dorsal skin distributed over 10 spots of 100 μl (one time only). Clinical signs were recorded by daily cage-side monitoring of behavioral changes (apathy, loss of appetite) or pain (avoidance of limb usage). Monkeys were sedated by intramuscular injection of 0.1 ml/kg of ketamine (10 mg/ml) for determination of bodyweight (an accepted surrogate disease marker for the CIA model), body temperature, blood collection and a physical inspection of the limbs for redness and/or swelling of the joints twice weekly. For the clinical and ethical management of the monkeys, observations were recorded using the integrated discomfort scoring scheme previously described [24-26].

To determine the efficacy of PDL241, groups were treated with either vehicle, PDL241 (30 mg/kg) or PDL241 (100 mg/kg). Eight animals per group ensured sufficient statistical power. The evaluation period was 70 days. Dosing solutions were given as a bolus infusion on days 7, 21 and 35. A planned fourth infusion on day 49 was cancelled due to the development of systemic infusion reactions in eight drug-treated animals (one death) shortly after the third infusion. We hypothesized that this infusion reaction was caused by the development of anti-drug antibodies (ADA) around day 35; therefore, a decision was made to cancel the fourth infusion. ADA were confirmed at the end of study using an ELISA-based method.

Overall clinical score, a composite score ranging from 0 to 5, was the primary endpoint. Serum C-reactive protein (CRP) levels, body weight loss, soft-tissue swelling (STS) count, serum levels of collagen-specific IgG and IgM, urinary excretion of collagen breakdown products hydroxylysylpyridinoline (HP) and lysylpyridinoline (LP) (biomarker of bone remodeling), histopathology and time to sacrifice were secondary endpoints. Following immunization, all monkeys developed an acute phase response (serum CRP level >50 mg/L after induction of arthritis), indicating that 100% of all animals showed characteristics of an ongoing severe inflammatory process. Urinary excretion of the collagen crosslinks HP and LP was determined twice weekly, starting from the day of CIA induction, as previously described [24,27]. The levels of HP and LP were normalized to creatinine levels (nmol levels per mmol creatinine) to compensate for a possible dilution by spilled drinking water. Blood markers of CIA were examined. Blood for hematology and for serum chemistry was collected once a week; CRP analysis was performed twice a week. All hematological and clinical chemistry analyses were performed at the Laboratory for Clinical Chemistry (BPRC) on a Sysmex Sf-3000 (Goffin Meyvis, The Netherlands) and a COBAS INTEGRA-400+ (Roche, Almere, The Netherlands), respectively. Serum samples were collected twice weekly for analyses of rhesus anti-chCII antibody levels of the IgM and IgG isotype as described elsewhere [28].

Histological parameters of the joint were examined. One proximal (PIP) and one distal interphalangeal (DIP) joint of one toe and finger of each foot and hand (two fingers/toes with outward signs of inflammation; two fingers/toes with no visible signs of inflammation) were processed at the BPRC for histopathological examination for synovitis and/or bone/cartilage destruction. After fixation in 4% phosphate-buffered formalin, the bones were decalcified for at least three weeks in Kristensen’s solution (17% formic acid in 1 *M* NaOH, pH 2.2). Decalcified bones were washed in tap water for 16 hours, dehydrated in ethanol/toluene, and embedded in paraffin. Sections of 2 μm thickness were cut and stained with hematoxilin/eosin. Histopathology was analyzed and graded by a pathologist blinded to the study. Histopathology was scored based on a histopathology grading system published by Pettit *et al.*[29]. This system quantifies the degree of inflammation, cartilage damage and bone damage on an arbitrary scale from 0 to 5.

### Statistical analysis

Due to the development of neutralizing ADA prior to day 35, followed by the subsequent loss of drug exposure, the data analysis was limited to the period from day 0 to day 31 post induction. Late responders to CIA induction (CRP levels >100 mg/l after day 21) may have experienced a limited effect of the treatment because of the previously described development of neutralizing antibodies. Analysis was, therefore, performed on ‘all animals’ (n = 8/group) and on those animals that responded early to the induction (CRP levels >100 mg/l on or before day 21; ‘early CRP onset group’; Placebo group n = 5; 30 mg/kg group n = 5; 100 mg/kg group n = 7). Statistical analyses were conducted using Prism 5 software (GraphPad Software, Inc. La Jolla, CA, USA). Statistical differences comparing the placebo-treated group at each time point with either treated group (30 mg/kg or 100 mg/kg) were determined using a two-tailed unpaired t test. Results with *P* <0.05 (*) or *P* <0.01 (**) were considered to be statistically significant.

## Results

### Expression of CD319 in RA synovium

To identify the immune cell subsets that co-express CD319 in RA synovium, FFPE synovial tissues from 26 RA subjects were stained with a mAb to CD319 (clone 1G9) and various hematopoietic cell markers. Expression of CD319 was restricted to infiltrating leukocytes (Figure 1A), with few cells double stained for CD319 and markers of T cells (CD3, Figure 1B), B cells (CD20, Figure 1C), NK cells (CD56, Figure 1D), or macrophages (CD68, Figure 1E). Figure 1E was taken from a portion of the tissue different than the other markers to obtain a clear visualization of the macrophages. The cells that were CD319^+^ were predominantly CD138^+^ plasma cells (Figure 1F). The expression pattern of CD319 in RA tissues, therefore, was different from that of the CD20 antigen recognized by rituximab, and provided the opportunity to directly target plasma cells.

**Figure 1:** **CD319 is expressed on RA synovial tissue (IHC) and is a marker of plasma cells.** FFPE samples of synovial tissues from RA patients were used for IHC analysis of CD319 using **(A)** 1G9 alone and co-stained with cell surface markers for leukocyte subsets **(B-F)**. Double labeling studies were performed using 1G9 in combination with **(B)** anti-CD3 (T cells), **(C)** anti-CD20 (B cells), **(D)** anti-CD56 (NK cells), **(E)** anti-CD68 (macrophages), and **(F)** CD138 for plasma cells. Brown staining represented CD319 reactivity while other cell surface markers stained red. Double staining cells are purple. FFPE, formalin fixed paraffin embedded; IHC, immunohistochemistry; RA, rheumatoid arthritis.

### PDL241 binding to leukocytes

The restricted expression of CD319 on RA synovium plasma cells prompted the generation of PDL241, a novel humanized mAb to CD319, as described in the Methods section. As there is disparate literature on the binding of anti-CD319 mAb to leukocytes, especially the binding to the B lymphocyte lineage [9,11,30-33], an extensive analysis of the binding of PDL241 to various leukocyte subsets from human blood was performed. PDL241 bound to the majority of NK cells, a subset of CD8^+^ T cells, a minor sub-population of CD4^+^ T cells, and plasmacytoid and myeloid DC but not naïve B cells, memory B cells, resting monocytes or granulocytes (Figure 2A). Binding of PDL241 to B cell subpopulations was specific for plasmablasts and plasma cells (described below). In addition, the binding of PDL241 on sections of normal human tonsil (a rich source of B lymphocytes that express a variety of phenotypes and activation states) was examined, and confirmed that PDL241 bound to VS38c^+^ plasma cells (Figure 2B).

**Figure 2:** **Binding of PDL241 to leukocytes. (A)** PBMC subsets were labeled for immunofluorescence analysis on the basis of co-staining: CD3+ CD4+ and CD3 + CD8+ (T cells); CD3-CD56+ (NK cells) and CD3 + CD56+ (NKT cells); CD19+ (B cells) and CD14+ (monocytes); CD27 + CD38 + CD138+ (plasmablasts and plasma cells). Lineage negative cells were first gated and then separated into HLA-DR + CD11c + (mDC), HLA-DR + CD123+ (pDC) and HLA-DR-CD123+ (basophils). Data representative of 1 of 10 donors. **(B)**  Immunofluorescence analysis of co-staining of PDL241 (green) with anti-CD3 (T cells), anti-CD20 (B cells) or VS38c Ab (plasma cells) in red on OCT embedded frozen tissues from normal human tonsil. Nuclei were counter-stained with DAPI (blue). Double stained cells appeared yellow. Ab, antibody; DAPI, 4′,6-diamidino-2-phenylindole; NK, natural killer; OCT, optimal cutting temperature; PBMC, peripheral blood mononuclear cells.

### Fc-dependent inhibition of Ig production by PDL241

The leukocyte subset binding pattern of PDL241 prompted the examination of the effect of the mAb in assays of B cell function. As PDL241 bound to terminally differentiated B cells, the activity of the mAb on the production of Ig by PWM-stimulated PBMC was examined. PDL241 was engineered with a human IgG_1_ Fc domain, and as a consequence, IgM was measured in the Ig production assays to limit interference from the humanized mAb. In time-course studies, a single high concentration (10 μg/ml) of PDL241 inhibited IgM measured in the supernatants of PBMC cultures seven days and nine days after initiation of the cultures (Figure 3A). The inhibition of PWM-induced IgM production by PDL241 was dependent on both the concentration of mAb and the presence of an intact Fc region, as PDL241 F(ab’)_2_ did not inhibit IgM production (Figure 3B). The ability of intact PDL241 but not F(ab’)_2_ PDL241 to inhibit IgM production was suggestive of a role for Fc receptors in the activity of PDL241. To identify an FcR-bearing cell subset responsible for mediating the activity of PDL241, NK cells or monocytes were depleted from PBMC by positive selection prior to the addition of PDL241. Depletion of NK cells but not monocytes greatly reduced the activity of PDL241 (Figure 3C). To determine if PDL241 inhibited Ig production by actively depleting B cells or plasma cells, the total number of live plasmablasts, B cells and T cells were determined after culture of PBMC with CpG and PDL241. In contrast to rituximab and consistent with the binding pattern of PDL241 to various B cell subsets, PDL241 had no effect on B cell counts (Figure 3D). However, both PDL241 and rituximab significantly reduced the number of plasmablasts. PDL241 and rituximab had no effect on T cell counts in these cultures. The activity of rituximab was likely due to the removal of resting B cells, which were therefore unable to differentiate into plasmablasts as CD20 is not expressed on plasmablasts and plasma cells [8]. To confirm the specificity of PDL241 for late stage, differentiated plasmablasts, PBMC were cultured for six days and the expression of CD319 on the CD27^+^CD38^+^ plasmablasts was measured. These cells were uniformly high for CD319 expression (Figure 3E). Addition of PDL241 to the cultures resulted in the disappearance of the CD319^hi^CD27^+^CD38^+^ cells. The data indicated that PDL241 mediated its inhibitory effect on IgM production by depleting CD319^+^ plasmablasts in an Fc-FcR-dependent manner.

**Figure 3:** **PDL241 inhibits Ig production from PBMC by specifically depleting plasmablasts and plasma cells. (A)** Time course of inhibition of IgM production from PBMC. Representative of n = 2 experiments. **(B)** Inhibition of IgM by PDL241 is dependent on mAb concentration and intact mAb, as F(ab’)2 fragments of PDL241 showed no activity. The dose dependent inhibition of IgM by PDL241 was demonstrated in >10 donors; F(ab’)2 experiment was a representative experiment of two. **(C)** Depletion of NK cells but not monocytes from PBMC reduces the inhibitory activity of PDL241. Representative experiment of n = 4; *P* = 0.01 for NK cell depleted compared to PBMC. **(D)** PDL241 treatment results in specific reduction in plasmablast counts in PBMC cultures. In contrast to rituximab (open bars), PDL241 treatment (closed bars) of PBMC specifically depleted plasma cells but not B cells from PBMC cultures. Counts were expressed as% of cIgG1-treated cultures. Data represent the mean and SD of n = 6 experiments from distinct donors. *P* ≤0.001 for B cell depletion by rituxan compared to PDL241 at 1 and 10 μg/ml. **(E)** CD319 was highly expressed on plasmablasts in PBMC cultures, (left panel, black histogram). Dot plots showing CD27 + CD38+ plasmablasts following treatment with cIgG1 control (middle panel) or PDL241 (right panel). Ig, immunoglobulin; mAB, monoclonal antibody; NK, natural killer; PBMC, peripheral blood mononuclear cells; SD, standard deviation.

### PBMC-RA synovial fibroblast co-culture

Given the strong expression of CD319 in leukocyte infiltrates in RA synovial tissue and the inhibitory activity of PDL241 on Ig production, the ability of PDL241 in modulating inflammatory cellular reactions within an RA lesion was modeled using a PBMC-RA synovial fibroblast (RASF) co-culture [34]. In this co-culture model, the direct cell contact interaction and/or the release of activating factors by RASF-activated B cells led to an increase in CD27^+^CD38^+^ plasmablasts/plasma cells. Consistent with the data described above, CD27^+^CD38^+^CD138^+^ plasma cells were positive for CD319, whereas CD27^+^CD38^-^ memory B cells and CD27^-^CD38^+^ naïve B cells were CD319^-^ (Figure 4A). Addition of PDL241 to the PBMC-RASF co-cultures specifically depleted the plasma cells, whereas rituximab depleted all B cell populations (Figure 4B). As rituximab does not bind to CD20^-^ plasma cells, it is likely that the effect of rituximab in these assays was due to depletion of cells prior to differentiation to plasma cells. An Fc-binding deficient mutant of PDL241 (241-G2M3) had no effect on cell depletion, confirming that the mechanism of depletion was Fc-FcR dependent.

**Figure 4:** **PDL241 treatment of RA synovial fibroblast-PBMC co-cultures leads to reduction on plasmablasts with no effect on B cells. (A)** B cells differentiated into CD19^+^CD27^hi^CD38^hi^CD319^+^ plasmablasts after co-culture with RA-synovial fibroblasts. PBMC from normal donors were cultured with RA synovial fibroblasts. At day 0 and day 7, cells in the culture were analyzed by flow cytometry. After co-culture for seven days, differentiated plasmablast cells (CD19^+^CD27^hi^CD38^hi^) (gate 1) could be detected and were found to be CD319 positive (solid line) as compared to isotype control staining (dotted line); in contrast, memory (CD19^+^CD27^+^) (gate 2) and naïve B cells (CD19^+^CD27^−^) (gate 3) did not express CD319. **(B)** Removal of CD319^+^ plasmablast cells by PDL241 in RA synovial fibroblast-PBMC co-cultures. Addition of PDL241 to cultures specifically depleted CD19^+^CD27^hi^CD38^hi^ plasmablasts, as compared to rituximab, which depleted only B cells. A FcR-binding deficient mutant of PDL241 (241-G2M3) had no effect on plasmablast cell numbers. The number in the gated population was calculated based on 10,000 events recoded. A representative experiment of n = 4 is shown. PBMC, peripheral blood mononuclear cells; RA, rheumatoic arthritis.

### CD319 expression and activity of PDL241 in HuSCID mice

To investigate the effect of PDL241 in an *in vivo* model, NSG mice were reconstituted with human PBMC and treated with PDL241. In preliminary experiments to verify human PBMC reconstitution, spleens of mice that had been transfused with human PBMC were harvested 14 days after initial cell injection for expression analysis. CD319 expression on human leukocytes in the spleens was confirmed by staining with human specific mAb 1G9. Double staining of 1G9 (green) and cell surface markers (red) was used to confirm CD319 expression on the engrafted human leukocytes. Cells of human origin were detected by staining for human CD45. Many human CD45+ leukocytes expressed CD319 (Figure 5A). Consistent with previous observations in normal human PBMC, almost all CD56^+^ NK cells and the majority of VS38c^+^ plasma cells in the mouse spleens were double stained indicating CD319 expression (yellow, Figure 5A). In contrast, very few CD3^+^ T cells or CD20^+^ B cells expressed CD319.

**Figure 5:** **PDL241 binds human leukocytes and inhibits human Ig production in huSCID mice.** NSG mice were transfused with human PBMC. **(A)** Double staining of CD319 (green fluorescence) and human leukocyte cell surface markers as indicated (red fluorescence) in the spleen. Cells expressing both markers were co-stained and appear yellow. 600X magnification. **(B)** Mice were sorted into groups on day 10 post-transfusion, and dosed twice weekly with PDL241 or cIgG1. IgM levels in the serum were measured at day 32 and day 47. In this experiment, PDL241 treatment resulted in significant reduction of human IgM compared to cIgG1 (day 32 *P* = 0.003 and day 47 *P* = 0.004 two tailed t-test). Significant reduction in IgM was observed in 6 of 11 separate experiments. huSCID, human-severe combined immunodeficiency; Ig, immunoglobulin; PBMC, peripheral blood mononuclear cells.

The presence of both human NK cells and CD319-expressing plasma cells provided the rationale to test the activity of PDL241 on human IgM production in this model. Detectable levels of human IgM on day 14 in the mouse sera ranged from 0 to 100 μg/ml, and treatment groups were block randomized from mice with serum concentrations of human IgM >10 μg/ml. Experiments in which a majority of mice had <10 μg/ml human IgM on day14 were terminated. Treatment groups were analyzed for the serum levels of human IgM post-treatment twice at approximately two week intervals. An example of a study showing significant activity of PDL241 on reducing human IgM levels is shown (Figure 5B). PDL241 significantly reduced the IgM levels in Hu-SCID sera in 6 of 11 experiments. The reason for the experiment-to-experiment variation in PDL241 activity is unclear, but may reflect the health of human FcR positive cells in the engrafted mice.

### Evaluation of PDL241 activity on biomarkers of CIA in rhesus monkeys

Since binding of PDL241 is restricted to human and non-human primate CD319 and does not bind to CD319 from rodent species, including mouse and rat (data not shown), the effect of treatment with PDL241 could not be evaluated in rodent models of arthritis. Therefore, a NHP model of arthritis (collagen-induced arthritis, CIA) was utilized. Disease symptoms in the rhesus monkey CIA model are critically dependent on anti-collagen type II (CII) immunoglobulins [22,25]. Given the effects of PDL241 on Ig production *in vitro* and in NSG mice, the hypothesis that PDL241 would reduce the severity of arthritic disease by inhibiting antibody production against CII was tested.

To ascertain that the CD319 expression pattern in rhesus monkeys was similar to that in humans, PDL241 was used to stain frozen sections from rhesus lymph node. PDL241 bound to VS38c^+^ plasma cells in rhesus monkey lymph node and tonsil, but not to CD20^+^ B cells (Figure 6A). In addition, CD319 was over-expressed in draining lymph nodes from rhesus monkeys that had been immunized with type II collagen and developed arthritic disease (Figure 6B). Functional analysis demonstrated that PDL241 was able to inhibit ODN2006-induced IgM production from rhesus PBMC, albeit with approximately 10 fold lower potency than for human PBMC (Figure 6C). This data is consistent with Surface Plasmon Resonance analysis showing that the binding affinity of PDL241 to rhesus CD319 was 10 to 20 fold lower than to human CD319. As observed in human PBMC cultures, the activity of PDL241 was dependent on Fc-FcR interactions as the FcR-binding deficient mAb 241-G2M3 had no activity in these assays.

**Figure 6:** **PDL241 binds to plasma cells in rhesus monkey. (A)** Immunofluorescence co-staining of PDL241 and anti-CD20 or VS38c in tonsils from normal rhesus monkey. PDL241 staining was green, CD20 and VS38c stained red and nuclei were counter-stained with DAPI (blue). Cells with double staining (PDL241 and VS38c) appeared yellow. **(B)** IHC staining of PDL241 to draining lymph nodes from normal (N) or collagen immunized (CIA) rhesus monkey. **(C)**. PDL241 but not Fc mutant 241-G2M3 inhibited IgM production from rhesus monkey PBMC stimulated with the TLR-9 agonist ODN2006. CIA, collagen-induced arthritis; DAPI, 4′,6-diamidino-2-phenylindole; IgM, immunoglobulin M; IHC, immunohistochemistry; PBMC, peripheral blood mononuclear cells.

A separate pharmacokinetics/pharmacodynamics (PK/PD) study in rhesus monkeys designed to identify the optimal dosing strategy to ensure sufficient occupancy of CD319 on peripheral lymphocytes by PDL241 over the 70 day study was conducted prior to the efficacy study in the CIA model. Simulation modeling suggested that a regimen of 30 mg/kg every two weeks (q2w) for a total of four doses would maintain a saturating serum concentration of PDL241 for 70 days. A high dose (100 mg/kg) group was included in order to maximize the pharmacological activity of PDL241. This dose was selected as the maximum amount of drug that could be infused based on the formulation. No major toxicities had been observed at this dose level in a separate non-GLP multiple dose-range finding study in cynomolgus monkeys (data not shown). A group of 24 healthy rhesus monkeys (male/female) were immunized with chicken type II collagen (chCII) emulsified in CFA. All 24 animals developed an acute phase response (CRP >50 mg/L after day 7) characteristic of an ongoing severe inflammatory process during the course of the study. In this model, the association between early onset of CRP in immunized monkeys with the rapid loss of body weight (and, therefore, a more rapid and severe form of the disease), has been established [26]. We also observed the development of a strong ADA response in the majority of monkeys treated with PDL241 (data not shown). ADA responses are common in NHP treated with humanized mAb due to the xenogenic nature of the human immunoglobulin. The consequence of ADA in this study was reduced exposure of the mAb, which decreased the ability of PDL241 at the doses administered to be effective at later time points (data not shown). To this end, efficacy data in this study were analyzed from all animals and in a subset of animals with early onset of CRP based on the time the serum CRP reached 100 mg/L after immunization (‘early CRP onset’). The subgroup analysis allowed the comparison of treatment versus placebo groups in monkeys that had a more rapid onset and severe disease while removing those monkeys with later disease onset from the analysis.

Treatment with PDL241 at 30 or 100 mg/kg had no or a minimal (not statistically significant) effect on all clinical parameters tested in analyses of all animals (Figure 7) or the early CRP onset subgroup (not shown). These parameters included bodyweight loss (Figure 7A), clinical score, (Figure 7B), increase in serum CRP (Figure 7C), onset of clinical symptoms (Figure 7D) and overall survival time (Figure 7E). Despite the lack of statistically significant activity on the clinical endpoints, a detailed investigation into the sub-clinical, joint-related, inflammatory responses was undertaken. The analysis of the early CRP onset subgroup (but not the all animals group) showed activity of PDL241 in alleviating these joint-related endpoints in the subgroup of monkeys with an early CRP onset. A dose-dependent decrease in the production of chCII specific IgM and IgG antibodies was observed in the ‘early CRP onset’ group (Figure 8A and B). The overall clinical score does not take into account the number of joints that are affected (joints with soft tissues swelling) and the severity of swelling for each individual joint. These parameters are summarized in the Small Joint Swelling Score (SJS, the sum of the severity of swelling for all arthritic small joints). A dose-dependent reduction in SJS was observed in the ‘early CRP onset’ groups treated with PDL 241 compared to the placebo treated group which attained statistical significance in the ‘early CRP onset’ animals treated with 100 mg/kg (Figure 8C). Along with an effect on anti-collagen antibodies and the SJS score, a decrease in damage to cartilage and bone in the early CRP onset group was inferred by the reduction in the collagen breakdown products HP (Figure 8D) and to a lesser extent with LP (Figure 8E) measured in the urine.

**Figure 7:** **PDL241 had no effect on clinical parameters in the rhesus monkey CIA model.** The analysis of all animals showed no effect of PDL241 on **(A)** bodyweight loss relative to day 0; **(B)** average clinical score; and **(C)** serum CRP levels. PDL241 treatment had no effect on **(D)** disease free survival or **(E)** overall survival. CIA, collagen-induced arthritis; CRP, C-reactive protein.

**Figure 8:** **PDL241 treatment reduced the severity of joint-related disease parameters in a rhesus CIA model.** Analyses are provided for ‘all animals’ and animals with ‘early CRP onset’ as described in the Methods section. Collagen type II-specific IgM **(A)** and IgG **(B)** were measured by ELISA. **(C)** The small joint swelling score is a representation of the number of joints affected (joints with soft tissues swelling) and the severity of swelling for each individual joint. Urinary excretion of the collagen crosslinks **(D)** hydroxylysylpyrridinoline (HP) and **(E)** lysylpyrridinoline (LP) was determined, with the levels normalized to creatinine levels (nmol levels per mmol creatinine) to compensate for a possible dilution by spilled drinking water. Pl = Placebo, 30 = 30 mg/kg and 100 = 100 mg/kg. * *P* ≤0.05; ** *P* ≤0.01. CIA, collagen-induced arthritis; CRP, C-reactive protein; Ig, immunoglobulin.

The effect of the treatment was also analyzed at the level of histopathology. In total, eight joints/animal (four PIPs and four DIPs; one finger/extremity) were analyzed for histopathology. Analysis of both the ‘all animals’ (Figure 9A) and the ‘early CRP onset’ subgroup (Figure 9B) showed a dose dependent reduction in inflammation, cartilage damage and bone damage that was highly significant for animals treated with 100 mg/kg.

**Figure 9:** **PDL241 treatment reduced the severity of joint-related histopathological parameters in the rhesus CIA model.** The histopathology score was based on a grading system described by Petit *et al*. [29]. Analyses were performed for **(A)** ‘all animal’ or **(B)** the ‘early CRP onset’ subgroup. CIA, collagen-induced arthritis; CRP, C-reactive protein.

## Discussion

The treatment paradigm for RA has changed significantly with the advent of biologic therapies, including inhibitors of TNF-α, costimulation blockade, CD20-mediated B cell depletion and modulation of the IL-6 pathway [35]. However, there remains a need to identify safe and effective treatments for patients refractory or intolerant to the current standard of care. In the current study, CD319 was identified as a potential therapeutic target using IHC analysis of RA synovial tissue, where the molecule was expressed at high levels on CD20 negative plasmablasts and plasma cells. The further differentiation of CD319 from CD20-targeted therapies was observed using PDL241, a novel humanized IgG_1_ mAb. PDL241 inhibited Ig production from PBMC *in vitro* by specifically depleting plasmablasts and plasma cells that expressed high levels of surface CD319, via antibody-dependent cellular cytotoxicity (ADCC). The activity of PDL241 in a rhesus monkey model of CIA provided further support as to the therapeutic potential of anti-CD319 therapy in RA. An anti-CD319 approach may provide particular benefit to patients who are refractory to anti-CD20 therapy with the presence of late stage plasmablasts in their disease tissue [7]. It is expected that PDL241 will show a different safety profile than anti-CD20 therapy due to the targeting of plasmablasts and plasma cells by PDL241. However, as B cells are thought to have a broader role in the autoimmune process, including antigen presentation, assisting in the development of lymphoid tissue architecture within the joint, and production of inflammatory cytokines [6], further investigation of CD319 biology in the RA disease process is warranted.

The mechanism of action of PDL241 is similar to that of another anti-CD319 mAb, elotuzumab. Elotuzumab has shown potent activity *in vitro* and *in vivo* against multiple myeloma cell lines and primary multiple myeloma cells, with the activity in both settings being attributed to ADCC. Neither PDL241 nor elotuzumab mediate complement dependent cytotoxicity or direct cytotoxic activity [36]. PDL241 binds a different epitope on CD319 than elotuzumab, with the PDL241 epitope residing on the membrane distal V domain, whereas elotuzumab binds the proximal C2-Ig domain. These mAb have differential effects on CD319 function. Elotuzumab enhances the homotypic adhesion of CD319, whereas PDL241 inhibits this interaction (Collins *et. al*., submitted). The role of CD319 as an ADCC target may come from its polarized expression in uropods [16]. Along with the ability to associate in a homotypic manner, CD319 has also been postulated to be involved in the interaction of multiple myeloma cells with bone marrow stroma [16]. The counter-receptor for CD319 on bone marrow stromal cells has not been defined, but is likely distinct from CD319, which has expression restricted to hematopoietic cells [9]. Although the function of CD319 on plasma cells is not known, it is possible that it plays a role in the bone marrow niches for plasma cell survival. Likewise, a role for CD319 in mediating interactions of leukocytes with the stroma in the inflamed synovium has not been investigated.

PDL241 showed promising activity in the rhesus monkey CIA model. The development of clinical arthritis in the CIA model is dependent on the production of CII specific IgM [28]. Mamu-B 26^-ve^ rhesus monkeys of Indian origin develop clinical arthritis and show a good production of CII specific IgM. Mamu-B 26^+ve^ rhesus monkeys are resistant to the development of clinical arthritis with heavily reduced serum levels of CII specific IgM [28]. Furthermore, the production of IgM is prominently associated with early responders to induction. The activity of PDL241 on anti-collagen antibodies observed in the model was consistent with the ability of the mAb to inhibit IgM production by PBMC *in vitro*. Although effects were detected on other disease-related parameters, there was a minimal effect on overall clinical scores, in part due to the severe inflammatory response in this model. Due to the labor-intensive nature of this model and only limited experience with other biologic drugs that are in the public domain [26], it was not possible to benchmark currently approved therapeutics in the current study.

The *in vivo* study was hampered by the immunogenicity of PDL241 in this rhesus monkey model, resulting in the development of ADA leading to strong infusion reactions following the third infusion. Retrospective analysis confirmed the presence of high levels of neutralizing ADA in serum collected on day 35 before the third infusion, and moderate to high levels of IL-6 and TNF-α were detected in serum collected shortly after infusion. A 90% reduction in complement levels (as determined by the CH50 assay) was also observed in post-dose serum samples (data not shown). As the reaction was observed at later time points and not associated with the initial dose of PDL241, it is likely that the infusion reactions were mediated by immunocomplexes of ADA and PDL241. A similar response to PDL241 was observed in a multiple dose GLP toxicology study, performed in parallel to this study in cynomolgus monkeys as part of the preclinical development of PDL241. Although ADA to human immunoglobulins in NHP are relatively common and not predictive of clinical immunogenicity [37], the magnitude of the response to PDL241 has prevented further development of this antibody. It is unclear if the strong immunogenicity of PDL241 was due to highly immunogenic amino acid sequences or the biology of the PDL241-CD319 interaction. The expression of CD319 on APC [11,38] may lead to enhanced presentation of humanized mAb leading to an enhanced ADA response. In support of this hypothesis, we have found that PDL241 was substantially more immunogenic in a huCD319 transgenic B57BL/6 mouse than in a wild-type B57BL/6 mouse (unpublished data). The association of CD319 with EAT-2 may also play a role in the enhanced immunogenicity of PDL241 [39].

Literature on the expression of CD319 on naïve B cells is not consistent, with studies showing no expression [9,11,33] and expression [30-32] on B cells prior to their activation and/or differentiation. PDL241 did not bind naïve B cells and did not deplete B cells in culture. There was no difference in the binding of PDL241 to the long or the short forms of CD319 when expressed on 293 cells (data not shown). The mAb used in IHC studies showed binding mainly to plasma cells in tissues with limited staining of other cell subsets (the current study, and [9]). As the sensitivity of IHC is lower than flow cytometry, the more limited expression pattern of CD319 in tissue was more likely a consequence of sensitivity rather than a reflection of different biology in tissues versus blood. The expression of CD319 on other leukocytes provides the potential for other mechanisms of action aside from the depletion of plasmablasts and plasma cells. CD319 expression has been reported on subsets of T cells, notably a subset of CD8+ T cells and activated CD4+ T cells, the majority of NK and NK T cells, DC and activated monocytes [9,11]. Binding of PDL241 was consistent with the published expression profile of CD319. The ability of PDL241 to inhibit T cell function was not examined in this study; however, preliminary data support an inhibitory activity on T cell proliferation via depletion of CD319-expressing T cells. The expression of CD319 on pDC and mDC [38] may provide further therapeutic opportunities for anti-CD319 mAb. Although development of PDL241 was halted due to the immunogenicity concerns described above, our data highlight the potential of CD319 as a therapeutic target in a range of autoimmune diseases where CD319-expressing cells have a role in the pathology.

## Conclusions

The expression of CD319 in RA synovium led to the investigation of the potential of CD319 as a target in RA. PDL241, a novel humanized mAb to CD319, demonstrated activity *in vitro* against plasmablasts/plasma cells and in a NHP model of RA. Our data highlight the therapeutic potential of targeting CD319, which may be especially relevant in anti-CD20 therapy non-responsive disease associated with the presence of plasmablasts.

## Abbreviations

ADA: Anti-drug antibodies; BPRC: Biomedical Research Research Centre; CFA: Complete Freund’s adjuvant; chCII: Chicken type II collagen; CIA: Collagen-induced arthritis; DAPI: 4′,6-diamidino-2-phenylindole; DC: Dendritic cells; DIP: Distal interphalangeal; ELISA: Enzyme-linked immunosorbent assay; FACS: Fluorescence-activated cell sorting; FPE: Formalin fixed paraffin embedded; HP: Hydroxylysylpyridinoline; hu-SCID: Human-severe combined immunodeficiency; Ig: Immunoglobulin; IHC: Immunohistochemistry; IL: Interleukin; ITSM: Immunoreceptor tyrosine-based switch motifs; LP: Lysylpyridinoline; mAb: Monoclonal antibody; NHP: Non-human primate; NK: Natural killer; NSG: NOD scid gamma chain knockout; OCT: Optimal cutting temperature; PBMC: Peripheral blood mononuclear cells; PBS: Phosphate-buffered saline; PIP: Proximal interphalangeal; RA: Rheumatoid arthritis; RF: Rheumatoid factor; SAP: SLAM-associated protein; SF: Synovial fibroblasts; SJS: Small joint swelling score; STS: Soft-tissue swelling; TNF: Tumor necrosis factor.

## Competing interests

JW, HK, DC, SY, JL, KL, IT, NB, TH, VV, DL and GS were employees of Facet Biotech, CA, which was acquired by AbbVie Inc. in 2010. Funding for this study was provided by Facet Biotech. AbbVie participated in the interpretation of data, review, and approval of the publication. MV, EB and BH declare that they have no competing interests.

## Authors’ contributions

JW designed the studies and wrote the manuscript; MV designed and performed NHP studies and wrote the manuscript; HK designed and performed *in vitro* studies; DC performed IHC analyses; SY, JL, KL and IT performed *in vitro* studies; NB performed mouse *in vivo* studies; TH participated in study design and produced PDL241; EB performed NHP studies; VV, BH and DL participated in study design, and GS designed the studies and wrote the manuscript. All authors read and approved the final manuscript.
